# The Synchronization Analysis of Cohen–Grossberg Stochastic Neural Networks with Inertial Terms

This article has been retracted.

**DOI:** 10.1155/2022/2377664

**Published:** 2022-05-25

**Authors:** Zhi-Ying Li, Wang-Dong Jiang, Yue-Hong Zhang

**Affiliations:** Yuanpei College of Shaoxing University, Shaoxing, Zhejiang, China

## Abstract

The exponential synchronization (ES) of Cohen–Grossberg stochastic neural networks with inertial terms (CGSNNIs) is studied in this paper. It is investigated in two ways. The first way is using variable substitution to transform the system to another one and then based on the properties of $i\hat{t}o$ integral, differential operator, and the second Lyapunov method to get a sufficient condition of ES. The second way is based on the second-order differential equation, the properties of calculus are used to get a sufficient condition of ES. At last, results of the theoretical derivation are verified by virtue of two numerical simulation examples.

## 1. Introduction

The dynamic behavior of neural network (NN) is a popular field in research studies and applications. Synchronization is one of the stability which has been studied a lot. Synchronization is the state in which two or more systems adjust their dynamic characteristics to achieve consistency under external driving or internal interaction.

In application, the external interference which can cause great uncertainty is everywhere, and the random interference is always inevitable. So, it is meaningful to consider stochastic term in the systems. The synchronization of stochastic neural networks has caught many scholars' attention. Li et al. studied the methodology to control the synchronization of stochastic system with memristive [1]. The ES of GSCGNNs is investigated by L Hu by graph-theory and state feedback control technique [2].

Synchronization of the systems is studied in [3–16] and so on. However, according to these research studies, the models considered do not contain inertial terms.

However, from the point of mathematics and physics, the model without inertial terms can be considered as the model of super damping, but when the damping surpasses the critical point, the dynamic properties of the neuron will change. So, it is meaningful to consider inertial terms in application. Li et al. analyzed the stability and synchronization of INNs delayed by generalized nonlinear measure approach and realized the quasi-synchronization by Halanary inequality and matrix measure (MM) [17]. Zhan et al. and Ke et al. studied the ES of inertial neural networks by using Lyapunov theory [18–20]. And there are other studies on the inertial neural networks [21–26].

So far, the neural networks on synchronization have been studied by adding only random terms in the system such as [1–16] or adding only inertial terms such as [17–26]. In application, the NN's dynamic behavior is not only disturbed by inertia (weak damping) but also influenced by random disturbance.

Therefore, it is meaningful to consider both of them in the systems. According to our enquiry, there is no result about synchronization containing both stochastic terms and inertial terms.

Motivated by the research studies above, the ES of CGSNNI is studied in this paper. The model is characterized by considering both stochastic factors and inertial factors. Two methods are used to obtain the ES. It will be a new topic and has its value in both theory and application.

This paper has an organization as follows: In section 1, the CGSNNI model is introduced. In section 2, preliminaries and lemmas are listed. In section 3, two theorems are proved. One is to transform the given second-order differential system into first-order by suitable variable substitution and then using differential operator and the second Lyapunov method to get a sufficient condition. The other one is derived from the second-order differential system, by using the properties of calculus. In section 4, two examples are simulated to verify the theorems. These two sufficient conditions derived are differently in the case of parameters given in the system and can complement each other.

We consider a class of CGSNNI as follows:

(1) $$\begin{array}{c} d\left({\dot{x}}_{i}\left(t\right)\right)=-\gamma_{i}{\dot{x}}_{i}\left(t\right)dt-\alpha_{i}\left(x_{i}\left(t\right)\right)\left[h_{i}\left(x_{i}\left(t\right)\right)-\sum_{j=1}^{n}a_{ij}f_{j}\left(x_{j}\left(t\right)\right)-I_{i}\left(t\right)\right]dt\\ +\sum_{i=1}^{n}c_{ij}g_{j}\left(x_{j}\left(t\right)\right)dB_{i}\left(t\right),\;i=1,2,\ldots ,n, \end{array}$$

where *t* ≥ 0, *x*_*i*_(*t*) is the state of the ith neuron at time *t*, *α*_*i*_(·) > 0 is the amplification function, *h*_*i*_(·) > 0 is the behavior function, *γ*_*i*_ > 0 is the damping coefficient, *a*_*ij*_ is the connection weights, *f*_*j*_(·) is the activation function of the jth neuron, *I*_*i*_(*t*) is the external input, and *B*(*t*)=(*B*_1_(*t*), *B*_2_(*t*),…,*B*_*n*_(*t*))^*T*^ is the *n* dimension Brown motion which is defined on complete probability space (Ω, *F*, Ρ), and *B*(*T*) has natural filtering {*F*_*t*_}_*t*≥0_.

Given the initial conditions of system (1) as follows:

(2) $$\begin{array}{c} \left\{\begin{array}{c} x_{i}\left(s\right)=\psi_{x_{i}}\left(s\right),\\ {\dot{x}}_{i}\left(s\right)=\chi_{x_{i}}\left(s\right), \end{array}s\leq 0,\right. \end{array}$$

where *ψ*_*x*_*i*__(*s*), *χ*_*x*_*i*__(*s*) are continuous.

Consider system (1) as the driven system, then the slave system of system (1) is as follows:

(3) $$\begin{array}{c} d\left({\dot{y}}_{i}\left(t\right)\right)=-\gamma_{i}{\dot{y}}_{i}\left(t\right)dt-\alpha_{i}\left(y_{i}\left(t\right)\right)\left[h_{i}\left(y_{i}\left(t\right)\right)-\sum_{j=1}^{n}a_{ij}f_{j}\left(y_{j}\left(t\right)\right)-I_{i}\left(t\right)\right]dt\\ +u_{i}\left(t\right)dt+\sum_{i=1}^{n}c_{ij}g_{j}\left({\text{y}}_{j}\left(t\right)\right)dB_{i}\left(t\right),i=1,2,\ldots ,n, \end{array}$$

where *u*(*t*)=(*u*_1_(*t*), *u*_2_(*t*),…,*u*_*n*_(*t*))^*T*^ is the control function.

Given the initial conditions of system (3) as

(4) $$\begin{array}{c} \left\{\begin{array}{c} y_{i}\left(s\right)=\psi_{y_{i}}\left(s\right),\\ {\dot{y}}_{i}\left(s\right)=\chi_{y_{i}}\left(s\right), \end{array}\right.s\leq 0, \end{array}$$

where *ψ*_*y*_*i*__(*s*), *χ*_*y*_*i*__(*s*) are continuous.

## 2. Preliminaries

The following assumptions are satisfied for *i*, *j*=1,2,…, *n*:

(*H*_1_) : *α*_*i*_(*x*_*i*_(*t*)) is bounded and derivable. That is, there exit constants ${\underline{\alpha }}_{i}>0,\bar{\alpha_{i}},A_{i}>0$, which satisfy
  (5) $$\begin{array}{c} {\underline{\alpha }}_{i}\leq \alpha_{i}\left(x_{i}\left(t\right)\right)\leq \bar{\alpha_{i}},\left|\alpha_{i}^{\prime }\left(x_{i}\right)\right|\leq A_{i}. \end{array}$$
(*H*_2_) : *f*_*j*_(·), *g*_*j*_(·) are bounded in *R* and satisfy Lipschitz conditions.
That is, there exit constants
  (6) $$\begin{array}{c} l_{j}>0,m_{j}>0,\bar{f_{j}}>0, \end{array}$$
which satisfy
  (7) $$\begin{array}{c} \left|f_{j}\left(u\right)-f_{j}\left(v\right)\right|\leq L_{j}\left|u-v\right|,\\ \left|g_{j}\left(u\right)-g_{j}\left(v\right)\right|\leq m_{j}\left|u-v\right|,\\ \left|f_{j}\left(\cdot \right)\right|\leq \bar{f_{j}},\;u,v\in R. \end{array}$$
(*H*_3_) : *k*_*i*_(*x*_*i*_)=*α*_*i*_(*x*_*i*_)*h*_*i*_(*x*_*i*_), *k*_*i*_(*x*_*i*_) is derivable, and there exist constants $\underline{k_{i}}>0,\bar{k_{i}}>0,$ which satisfy $0\leq \underline{k_{i}}\leq k_{i}^{\prime }\left(x_{i}\right)\leq \bar{k_{i}}.$

**Definition 1 .**

If there are constants *λ* > 0, *c* > 0, which satisfy

(8) $$\begin{array}{c} \sum_{i=1}^{n}E\left[{\left(x_{i}\left(t\right)-y_{i}\left(t\right)\right)}^{2}\right]\leq ce^{-\lambda \left(t-t_{0}\right)},\;t\geq t_{0}, \end{array}$$

then the drive system (1) and the slave system (3) are ES under the control strategy *u*(*t*).

**Lemma 1 .**

(see [27]).

(9) $$\begin{array}{c} \left\{\begin{array}{c} dx\left(t\right)=f\left(t,x\left(t\right)\right)dt+g\left(t,x\left(t\right)\right)dW\left(t\right),\;t\geq 0,\\ x\left(t_{0}\right)=x_{0.}, \end{array}\right. \end{array}$$

where *f* ∈ [*R*_+_ × *R*^*n*^, *R*^*n*^] and *g* ∈ [*R*_+_ × *R*^*n*^, *R*^*n*×*n*^] are functions which are Borel measurable and *W*(*t*) is the standard Brown motion in *R*^*n*^. We define a differential operator as follows:

(10) $$\begin{array}{c} L=\frac{\partial }{\partial t}+\sum_{j=1}^{n}f_{j}\left(t,x\right)\frac{\partial }{\partial x_{j}}+\frac{1}{2}\sum_{j=1}^{n}{\left[g\left(t,x\right)g^{T}\left(t,x\right)\right]}_{ij}\frac{\partial^{2}}{\partial x_{i}\partial x_{j}}. \end{array}$$

If *V*(*t*, *x*) ∈ *C*^1,2^[*R*_+_ × *S*_*h*_, *R*_+_], then

(11) $$\begin{array}{c} \text{LV}\left(t,x\right)=\frac{\partial V\left(t,x\right)}{\partial t}+\frac{\partial V\left(t,x\right)}{\partial x}f\left(t,x\right)+\frac{1}{2}\text{trace}{\left[g^{T}\left(t,x\right)\frac{\partial^{2}V\left(t,x\right)}{\partial x\;\partial x}g\left(t,x\right)\right]}_{ij}, \end{array}$$

where *S*_*h*_={*x|*‖*x*‖ ≤ *h*} ∈ *R*^*n*^,

(12) $$\begin{array}{c} \frac{\partial V}{\partial x}=\left(\frac{\partial V}{\partial x_{1}},\frac{\partial V}{\partial x_{2}},\ldots ,\frac{\partial V}{\partial x_{n}}\right),\frac{\partial^{2}V}{\partial x\;\partial x}={\left(\frac{\partial^{2}V}{\partial x_{i}\partial x_{j}}\right)}_{n\times n}. \end{array}$$

By $I\hat{t}o$ formula, if *x*(*t*) ∈ *S*_*h*,_ then

(13) $$\begin{array}{c} dV\left(t,x\left(t\right)\right)=LV\left(t,x\left(t\right)\right)dt+\frac{\partial V\left(t,x\right)}{\partial x}g\left(t,x\left(t\right)\right)dW\left(t\right). \end{array}$$

Under the substitutions,

(14) $$\begin{array}{c} z_{i}\left(t\right)={\dot{x}}_{i}\left(t\right)+\eta_{i}x_{i}\left(t\right),\eta_{i}>0,\;i=1,2,\ldots ,n. \end{array}$$

System (1) and system (2) are transformed into

(15) $$\begin{array}{c} \left\{\begin{array}{c} d\left(x_{i}\left(t\right)\right)=\left(-\eta_{i}x_{i}\left(t\right)+z_{i}\left(t\right)\right)dt\\ d\left(z_{i}\left(t\right)\right)=\eta_{i}\left(\eta_{i}-\gamma_{i}\right)x_{i}\left(t\right)dt-\left(\gamma_{i}-\eta_{i}\right)z_{i}\left(t\right)dt-\alpha_{i}\left(x_{i}\left(t\right)\right)\left[h_{i}\left(x_{i}\left(t\right)\right)\right.\\ -\sum_{j=1}^{n}a_{ij}f_{j}\left(x_{j}\left(t\right)\right)-I_{i}\left.\left(t\right)\right]dt+\sum_{j=1}^{n}c_{ij}g_{j}\left(x_{j}\left(t\right)\right)dB\left(t\right), \end{array}\right.\\ \left\{\begin{array}{c} x_{i}\left(s\right)=\psi_{x_{i}}\left(s\right),{\dot{x}}_{i}\left(s\right)=\chi_{x_{i}}\left(s\right),\\ z_{i}\left(s\right)=\eta_{i}\psi_{x_{i}}\left(s\right)+\chi_{x_{i}}\left(s\right). \end{array}\right. \end{array}$$

Take the substitutions

(16) $$\begin{array}{c} \omega_{i}\left(t\right)={\dot{y}}_{i}\left(t\right)+\eta_{i}y_{i}\left(t\right),\;\eta_{i}>0,\;i=1,2,\ldots ,n. \end{array}$$

One sees that system (3) and (4) are transformed into

(17) $$\begin{array}{c} d\left(y_{i}\left(t\right)\right)=\left(-\eta_{i}y_{i}\left(t\right)+\omega_{i}\left(t\right)\right)dt,i=1,2,\ldots ,n,\\ d\left(\omega_{i}\left(t\right)\right)=-\eta_{i}\left(\eta_{i}-\gamma_{i}\right)y_{i}\left(t\right)dt-\left(\gamma_{i}-\eta_{i}\right)\omega_{i}\left(t\right)dt-\alpha_{i}\left(y_{i}\left(t\right)\right)\left[h_{i}\left(y_{i}\left(t\right)\right)\right.\\ -\sum_{j=1}^{n}a_{ij}f_{j}\left(y_{j}\left(t\right)\right)-I_{i}\left.\left(t\right)\right]dt+u_{i}\left(t\right)dt+\sum_{j=1}^{n}c_{ij}g_{j}\left(y_{j}\left(t\right)\right)dB_{i}\left(t\right),\\ y_{i}\left(s\right)=\psi_{y_{i}}\left(s\right),{\dot{y}}_{i}\left(s\right)=\chi_{y_{i}}\left(s\right),\\ \omega_{i}\left(s\right)=\eta_{i}\psi_{y_{i}}\left(s\right)+\chi_{y_{i}}\left(s\right). \end{array}$$

Define the synchronization errors:

(18) $$\begin{array}{c} \nu_{1i}\left(t\right)=y_{i}\left(t\right)-x_{i}\left(t\right),\nu_{2i}\left(t\right)=\omega_{i}\left(t\right)-z_{i}\left(t\right). \end{array}$$

And let the control strategy be

(19) $$\begin{array}{c} u_{i}\left(t\right)=-\pi_{i}\nu_{1i}\left(t\right),\;\pi_{i}>0. \end{array}$$

From (1) and (3), one sees that

(20) dν1it=−ηiν1it+ν2itdtdν2it=−ηi2−ηiγi+πiν1itdt−γi−ηiν2itdt−αiyithiyit−αixithixitdt+αiyit∑j=1naijfjyit−fjxitdt+αiyit−αixit∑j=1naijfjxjt+Iitdt+∑j=1ncijgjyjt−gjxjtdBti,i=1,2,...,n.

## 3. Main Results

In this part, by using the properties of $i\hat{t}o$ integral, differential operator, and stability theory of Lyapunov and the properties of calculus, two sufficient conditions for the ES of CGSNNI are derived.

**Theorem 1 .**

In system (1), if (*H*_1_) − (*H*_3_) are satisfied, *I*_*i*_(*t*) is bounded, which means there exits *I*_*i*_ > 0 and *π*_i_ > 0, which satisfies |*I*_*i*_(*t*)| ≤ *I*_*i*_, and let the control strategy be

(21) $$\begin{array}{c} u_{i}\left(t\right)=-\pi_{i}\left(y_{i}\left(t\right)-x_{i}\left(t\right)\right). \end{array}$$

If

(22) $$\begin{array}{c} p_{i}=2\eta_{i}-\gamma_{i}\eta_{i}-r_{i}-\sum_{j=1}^{n}{\bar{\alpha }}_{j}\left|a_{ji}\right|l_{i}-\sum_{k=1}^{n}\sum_{j=1}^{n}c_{kj}^{2}m_{i}^{2}>0,\\ q_{i}=2\left(\gamma_{i}-\eta_{i}\right)-\gamma_{i}\eta_{i}-r_{i}-\sum_{j=1}^{n}{\bar{\alpha }}_{i}\left|a_{ij}\right|l_{j}>0, \end{array}$$

where $r_{i}=\left|1+\eta_{i}^{2}-\pi_{i}\right|+{\bar{k}}_{i}+A_{i}\sum_{i=1}^{n}\left|a_{ij}\right|{\bar{f}}_{j}+A_{i}I_{i},$*i*=1,2,…, *n* then the drive system (1) and the slave system (3) are ES under the control strategy *u*(*t*).

**Proof of Theorem 1.**

Let

(23) $$\begin{array}{c} \nu \left(t\right)={\left(\nu_{11}\left(t\right),\nu_{12}\left(t\right),\ldots ,\nu_{1n}\left(t\right),\nu_{21}\left(t\right),\nu_{22}\left(t\right),\ldots ,\nu_{2n}\left(t\right)\right)}^{T}, \end{array}$$

for any *ε* > 0, define a Lyapunov function as follows:

(24) $$\begin{array}{c} V\left(t,\nu \left(t\right)\right)=\sum_{i=1}^{n}e^{\varepsilon t}\left(\nu_{1i}^{2}\left(t\right)+\nu_{2i}^{2}\left(t\right)\right). \end{array}$$

One can see that

(25) $$\begin{array}{c} V_{t}\left(t,\nu \left(t\right)\right)=\sum_{i=1}^{n}e^{\varepsilon t}\varepsilon \left(\nu_{1i}^{2}\left(t\right)+\nu_{2i}^{2}\left(t\right)\right),\\ V_{\nu \left(t\right)}\left(t,\nu \left(t\right)\right)=2e^{\varepsilon t}\nu \left(t\right),\\ V_{\nu \left(t\right)\nu \left(t\right)}\left(t,\nu \left(t\right)\right)=2e^{\varepsilon t}E_{2n\times 2n}, \end{array}$$

where *E*_2*n*×2*n*_ is the 2*n* × 2*n* order identity matrix, and *V*_*v*(*t*)_(*t*, *v*(*t*)), *V*_*v*(*t*)*v*(*t*)_(*t*, *v*(*t*)) is the first and second derivatives with respect to *v*(*t*).

From Lemma 1 and (20),

(26) $$\begin{array}{c} \text{LV}\left(t,\nu \left(t\right)\right)=\sum_{i=1}^{n}\nu_{1i}\left(t\right)e^{\varepsilon t}\left\{\varepsilon \left(\nu_{1i}^{2}\left(t\right)+\nu_{2i}^{2}\left(t\right)\right)+2\left(-\eta_{i}\nu_{1i}\left(t\right)+\nu_{2i}\left(t\right)\right)\right.\\ -2\nu_{2i}\left(t\right)\left[\left(-\eta_{i}^{2}-\gamma_{i}\eta_{i}+\pi_{i}\right)\nu_{1i}\left(t\right)+\left(\gamma_{i}-\eta_{i}\right)\nu_{2i}\left(t\right)\right]\\ -2\nu_{2i}\left(t\right)\left[\alpha_{i}\left(y_{i}\left(t\right)\right)h_{i}\left(y_{i}\left(t\right)\right)-\alpha_{i}\left(x_{i}\left(t\right)\right)h_{i}\left(x_{i}\left(t\right)\right)\right]\\ +2\nu_{2i}\left(t\right)\alpha_{i}\left(y_{i}\left(t\right)\right)\sum_{j=1}^{n}a_{ij}\left(f_{j}\left(y_{j}\left(t\right)\right)-f_{j}\left(x_{j}\left(t\right)\right)\right)\\ +2\nu_{2i}\left(t\right)\left(\alpha_{i}\left(y_{i}\left(t\right)\right)-\alpha_{i}\left(x_{i}\left(t\right)\right)\right)\left[\sum_{j=1}^{n}a_{ij}f_{j}\left(x_{j}\left(t\right)\right)+I_{i}\left(t\right)\right]\\ \left.+{\left[\sum_{\text{i}=1}^{\text{n}}{\text{c}}_{\text{ij}}\left(g_{j}\left(y_{j}\left(t\right)\right)-g_{j}\left(x_{j}\left(t\right)\right)\right)\right]}^{2}\right\}. \end{array}$$

As (*H*_1_) − (*H*_3_) are satisfied, one can see that

(27) $$\begin{array}{c} \alpha_{i}\left(y_{i}\left(t\right)\right)-\alpha_{i}\left(x_{i}\left(t\right)\right)=\alpha_{i}^{\prime }\left(\xi_{i}\left(t\right)\right)\left(y_{i}\left(t\right)-x_{i}\left(t\right)\right),\\ k_{i}\left(y_{i}\left(t\right)\right)-k_{i}\left(x_{i}\left(t\right)\right)=\alpha_{i}\left(y_{i}\left(t\right)\right)h_{i}\left(y_{i}\left(t\right)\right)-\alpha_{i}\left(x_{i}\left(t\right)\right)h_{i}\left(x_{i}\left(t\right)\right)=k_{i}^{\prime }\left(\xi_{i}^{*}\left(t\right)\right)\left(y_{i}\left(t\right)-x_{i}\left(t\right)\right), \end{array}$$

where *ξ*_*i*_(*t*) and *ξ*_*i*_^*∗*^(*t*) are between *y*_*i*_(*t*) and *x*_*i*_(*t*).

Derive from (26),

(28) $$\begin{array}{c} \text{LV}\left(t,\nu \left(t\right)\right)\leq \sum_{i=1}^{n}e^{\varepsilon t}\left\{\varepsilon \left(\nu_{1i}^{2}\left(t\right)+\nu_{2i}^{2}\left(t\right)\right)+2\left(-\eta_{i}\nu_{1i}^{2}\left(t\right)+\nu_{1i}\left(t\right)\nu_{2i}\left(t\right)\right)\right.\\ -2\left(-\eta_{i}^{2}-\gamma_{i}\eta_{i}+\pi_{i}\right)\nu_{1i}\left(t\right)\nu_{2i}\left(t\right)+\left(\gamma_{i}-\eta_{i}\right)\nu_{2i}^{2}\left(t\right)\\ +2{\bar{k}}_{i}\left|\nu_{1i}\left(t\right)\right|\left|\nu_{2i}\left(t\right)\right|+2{\bar{\alpha }}_{i}\sum_{j=1}^{n}a_{ij}l_{j}\left|\nu_{1i}\left(t\right)\right|\left|\nu_{2i}\left(t\right)\right|\\ +2A_{i}\left|\nu_{1i}\left(t\right)\right|\left|\nu_{2i}\left(t\right)\right|\left[\sum_{j=1}^{n}a_{ij}{\bar{f}}_{j}+I_{i}\left(t\right)\right]+\left.{\left[\sum_{j=1}^{n}\left|c_{ij}\right|m_{j}\nu_{1j}\left(t\right)\right]}^{2}\right\}\\ \leq \sum_{i=1}^{n}e^{\varepsilon t}\left\{\left[\varepsilon -2\eta_{i}+\sum_{k=1}^{n}\sum_{j=1}^{n}c_{kj}^{2}m_{i}^{2}\right]\right.\nu_{1i}^{2}\left(t\right)\\ -\left(\varepsilon +2\gamma_{i}-2\eta_{i}\right)\nu_{2i}^{2}\left(t\right)+2\left(1+\eta_{i}^{2}+\gamma_{i}\eta_{i}-\pi_{i}\right)\nu_{1i}\left(t\right)\nu_{2i}\left(t\right)\\ +2\left[{\bar{k}}_{i}+A_{i}\sum_{j=1}^{n}\left|a_{ij}\right|{\bar{f}}_{j}+A_{i}I_{i}\right]\left|\nu_{1i}\left(t\right)\right|\left|\nu_{2i}\left(t\right)\right|\\ \left.+2{\bar{\alpha }}_{i}\sum_{j=1}^{n}\left|a_{ij}\right|l_{j}\left|\nu_{1j}\left(t\right)\right|\left|\nu_{2i}\left(t\right)\right|\right\}\\ \leq \sum_{i=1}^{n}e^{\varepsilon t}\left\{\left[\varepsilon -2\eta_{i}+\gamma_{i}\eta_{i}+\left|1+\eta_{i}^{2}-\pi_{i}\right|+{\bar{k}}_{i}+A_{i}\sum_{j=1}^{n}\left|a_{ij}\right|\right.\right.{\bar{f}}_{j}\\ +A_{i}I_{i}+\sum_{j=1}^{n}{\bar{\alpha }}_{j}\left|a_{ji}\right|l_{i}+\left.\sum_{k=1}^{n}\sum_{j=1}^{n}c_{kj}^{2}m_{i}^{2}\right]\nu_{1i}^{2}\left(t\right)\\ +\left[\varepsilon -2\gamma_{i}+2\eta_{i}+\gamma_{i}\eta_{i}+\left|1+\eta_{i}^{2}-\pi_{i}\right|+{\bar{k}}_{i}\right.\\ +A_{i}\sum_{j=1}^{n}\left|a_{ij}\right|{\bar{f}}_{j}+A_{i}I_{i}+\left.\sum_{j=1}^{n}{\bar{\alpha }}_{j}\left|a_{ij}\right|l_{j}\right]\left.\nu_{2i}^{2}\left(t\right)\right\}. \end{array}$$

According to the conditions in Theorem 1, if there exits *ε* > 0, which satisfy

(29) $$\begin{array}{c} \varepsilon -2\eta_{i}+\gamma_{i}\eta_{i}+\left|1+\eta_{i}^{2}-\pi_{i}\right|+{\bar{k}}_{i}+A_{i}\sum_{j=1}^{n}\left|a_{ij}\right|{\bar{f}}_{j}+A_{i}I_{i}+\sum_{j=1}^{n}{\bar{\alpha }}_{j}\left|a_{ji}\right|l_{i}+\sum_{k=1}^{n}\sum_{j=1}^{n}c_{kj}^{2}m_{i}^{2}\leq 0,\\ \varepsilon -2\gamma_{i}+2\eta_{i}+\gamma_{i}\eta_{i}+\left|1+\eta_{i}^{2}-\pi_{i}\right|+{\bar{k}}_{i}+A_{i}\sum_{j=1}^{n}\left|a_{ij}\right|{\bar{f}}_{j}+A_{i}I_{i}+\sum_{j=1}^{n}{\bar{\alpha }}_{j}\left|a_{ij}\right|l_{j}\leq 0. \end{array}$$

From that one has

(30) $$\begin{array}{c} \text{LV}\left(t,\nu \left(t\right)\right)\leq 0. \end{array}$$

In addition,

(31) $$\begin{array}{c} dV\left(t,\nu \left(t\right)\right)=\text{LV}\left(t,\nu \left(t\right)\right)dt+\frac{\partial V\left(t,\nu \left(t\right)\right)}{\partial \nu \left(t\right)}\left(g\left(y\left(t\right)\right)-g\left(x\left(t\right)\right)\right)dB\left(t\right),\\ V\left(t,\nu \left(t\right)\right)=V\left(0,\nu \left(0\right)\right)+\int_{0}^{t}\text{LV}\left(s,\nu \left(s\right)\right)\text{d}s\\ +2\int_{0}^{t}\sum_{i=1}^{n}\sum_{j=1}^{n}c_{ij}\nu_{2i}\left(s\right)\left(g_{j}\left(y_{j}\left(s\right)\right)-g_{j}\left(x_{j}\left(s\right)\right)\right)dB_{i}\left(s\right). \end{array}$$

As

(32) $$\begin{array}{c} V\left(t,\nu \left(t\right)\right)=\sum_{i=1}^{n}e^{\varepsilon t}\left(\nu_{1i}^{2}\left(t\right)+\nu_{2i}^{2}\left(t\right)\right), \end{array}$$

and LV(*t*, *ν*(*t*)) ≤ 0, one sees that

(33) $$\begin{array}{c} \sum_{i=1}^{n}\left(\nu_{1i}^{2}\left(t\right)+\nu_{2i}^{2}\left(t\right)\right)\leq e^{-\varepsilon t}\sum_{i=1}^{n}\left(\nu_{1i}^{2}\left(0\right)+\nu_{2i}^{2}\left(0\right)\right)+2e^{-\varepsilon t}\int_{0}^{t}\sum_{i=1}^{n}\sum_{j=1}^{n}c_{ij}\nu_{2i}\left(s\right)\left(g_{j}\left(y_{j}\left(s\right)\right)-g_{j}\left(x_{j}\left(s\right)\right)\right)\text{d}B_{i}\left(s\right). \end{array}$$

By taking expectations,

(34) $$\begin{array}{c} \sum_{i=1}^{n}E\left[\nu_{1i}^{2}\left(t\right)+\nu_{2i}^{2}\left(t\right)\right]\leq e^{-\varepsilon t}\sum_{i=1}^{n}E\left[\nu_{1i}^{2}\left(0\right)+\nu_{2i}^{2}\left(0\right)\right]. \end{array}$$

Therefore,

(35) $$\begin{array}{c} \sum_{i=1}^{n}E\left[\nu_{1i}^{2}\left(t\right)+\nu_{2i}^{2}\left(t\right)\right]\leq ce^{-\varepsilon t},\varepsilon >0,c>0,t\geq 0, \end{array}$$

where

(36) $$\begin{array}{c} c=\sum_{i=1}^{n}E\left[\nu_{1i}^{2}\left(0\right)+\nu_{2i}^{2}\left(0\right)\right]. \end{array}$$

It comes to

(37) $$\begin{array}{c} \sum_{i=1}^{n}E\left[{\left(x_{i}\left(t\right)-y_{i}\left(t\right)\right)}^{2}\right]\leq ce^{-\varepsilon t},\;\varepsilon >0,\;c>0,\;t\geq 0. \end{array}$$

According to Definition 1, system (1) and system (3) are ES under the control strategy *u*(*t*).

**Theorem 2 .**

If (*H*_1_) − (*H*_3_) are satisfied, *I*_*i*_(*t*) is bounded; that is, there exit *I*_*i*_ > 0 and *π*_i_ > 0, which satisfy |*I*_*i*_(*t*)| ≤ *I*_*i*_; let the control strategy be *u*_*i*_(*t*)=−*π*_*i*_(*y*_*i*_(*t*) − *x*_*i*_(*t*)).

If

(38) $$\begin{array}{c} 2\pi_{i}-\left|2-\gamma_{i}-\pi_{i}\right|-3{\bar{k}}_{i}-{\bar{\alpha }}_{i}\sum_{j=1}^{n}\left|a_{ij}\right|l_{j}-3A_{i}\left(\sum_{j=1}^{n}\left|a_{ij}\right|{\bar{f}}_{j}+I_{i}\right)>0,\\ 2\gamma_{i}-2-\left|2-\gamma_{i}-\pi_{i}\right|-{\bar{k}}_{i}-\sum_{j=1}^{n}{\bar{\alpha }}_{j}\left|a_{ji}\right|l_{i}-\sum_{j=1}^{n}{\bar{\alpha }}_{i}\left|a_{ij}\right|l_{j}-A_{i}\left(\sum_{j=1}^{n}\left|a_{ij}\right|{\bar{f}}_{j}+I_{i}\right)>0, \end{array}$$

then the drive system (1) and the slave system (3) are ES under control strategy *u*(*t*).

**Proof of Theorem 2.**

Let

(39) $$\begin{array}{c} \nu_{i}\left(t\right)=y_{i}\left(t\right)-x_{i}\left(t\right). \end{array}$$

From (1) and (3),

(40) $$\begin{array}{c} d\left({\dot{\nu }}_{i}\left(t\right)\right)=-\gamma_{i}{\dot{\nu }}_{i}\left(t\right)dt-\pi_{i}\nu_{i}\left(t\right)dt-\left[\alpha_{i}\left(y_{i}\left(t\right)\right)h_{i}\left(y_{i}\left(t\right)\right)-\alpha_{i}\left(x_{i}\left(t\right)\right)h_{i}\left(x_{i}\left(t\right)\right)\right]dt\\ +\alpha_{i}\left(y_{i}\left(t\right)\right)\sum_{j=1}^{n}a_{ij}\left[f_{j}\left(y_{j}\left(t\right)\right)-f_{j}\left(x_{j}\left(t\right)\right)\right]dt\\ +\left[\alpha_{i}\left(y_{i}\left(t\right)\right)-\alpha_{i}\left(x_{i}\left(t\right)\right)\right]\left[\sum_{j=1}^{n}a_{ij}f_{j}\left(x_{j}\left(t\right)\right)+I_{i}\left(t\right)\right]dt\\ +\sum_{j=1}^{n}c_{ij}\left[g_{j}\left(y_{j}\left(t\right)\right)-g_{j}\left(x_{j}\left(t\right)\right)\right]dB_{i}\left(t\right),i=1,2,\ldots ,n. \end{array}$$

For any *ε* > 0,

(41) $$\begin{array}{c} V\left(t\right)=\sum_{i=1}^{n}\left[\nu_{i}^{2}\left(t\right)+{\left(\nu_{i}\left(t\right)+{\dot{\nu }}_{i}\left(t\right)\right)}^{2}\right]e^{\varepsilon t}. \end{array}$$

From the two formulas above,

(42) $$\begin{array}{c} dV\left(t\right)=\sum_{i=1}^{n}\left\{\varepsilon \left[\nu_{i}^{2}\left(t\right)+{\left(\nu_{i}\left(t\right)+{\dot{\nu }}_{i}\left(t\right)\right)}^{2}\right]\right.e^{\varepsilon t}dt\\ \left.+2\left[\nu_{i}\left(t\right){\dot{\nu }}_{i}\left(t\right)+\left(\nu_{i}\left(t\right)+{\dot{\nu }}_{i}\left(t\right)\right)\left({\dot{\nu }}_{i}\left(t\right)+{\ddot{\nu }}_{i}\left(t\right)\right)\right]e^{\varepsilon t}dt\right\}\\ =e^{\varepsilon t}\sum_{i=1}^{n}\left\{\varepsilon \left[\nu_{i}^{2}\left(t\right)+{\left(\nu_{i}\left(t\right)+{\dot{\nu }}_{i}\left(t\right)\right)}^{2}\right]\right.dt\\ +2\nu_{i}\left(t\right){\dot{\nu }}_{i}\left(t\right)+2\left(\nu_{i}\left(t\right)+{\dot{\nu }}_{i}\left(t\right)\right){\dot{\nu }}_{i}\left(t\right)\\ +2\left(\nu_{i}\left(t\right)+{\dot{\nu }}_{i}\left(t\right)\right)\left\{-\gamma_{i}\right.{\dot{\nu }}_{i}\left(t\right)dt-\pi_{i}\nu_{i}\left(t\right)dt\\ -\left[\alpha_{i}\left(y_{i}\left(t\right)\right)h_{i}\left(y_{i}\left(t\right)\right)-\alpha_{i}\left(x_{i}\left(t\right)\right)h_{i}\left(x_{i}\left(t\right)\right)\right]dt\\ +\alpha_{i}\left(y_{i}\left(t\right)\right)\sum_{j=1}^{n}a_{ij}\left[f_{j}\left(y_{j}\left(t\right)\right)-f_{j}\left(x_{j}\left(t\right)\right)\right]dt\\ +\left[\alpha_{i}\left(y_{i}\left(t\right)\right)-\alpha_{i}\left(x_{i}\left(t\right)\right)\right]\left[\sum_{j=1}^{n}a_{ij}f_{j}\left(x_{j}\left(t\right)\right)+I_{i}\left(t\right)\right]dt\\ +\sum_{j=1}^{n}c_{ij}\left[g_{j}\left(y_{j}\left(t\right)\right)-g_{j}\left(x_{j}\left(t\right)\right)\right]\left.\left.dB_{i}\left(t\right)\right\}\right\}. \end{array}$$

Integral both sides by *t*,

(43) $$\begin{array}{c} V\left(t\right)\leq V\left(0\right)+\sum_{i=1}^{n}\int_{0}^{t}e^{\varepsilon s}\left\{\left(2\varepsilon -2\pi_{i}\right)\nu_{i}^{2}\left(s\right)+\left(\varepsilon +2-2\gamma_{i}\right){\dot{\nu }}_{i}^{2}\left(s\right)\right.\\ +\left(2\varepsilon +4-2\gamma_{i}-2\pi_{i}\right)\nu_{i}\left(s\right){\dot{\nu }}_{i}\left(s\right)+2{\bar{k}}_{i}\left(\left|\nu_{i}\left(s\right)\right|+\left|{\dot{\nu }}_{i}\left(s\right)\right|\right)\left|\nu_{i}\left(s\right)\right|\\ +2\left(\left|\nu_{i}\left(s\right)\right|+\left|{\dot{\nu }}_{i}\left(s\right)\right|\right){\bar{\alpha }}_{i}\sum_{j=1}^{n}\left|a_{ij}\right|l_{j}\left|{\dot{\nu }}_{j}\left(s\right)\right|\\ +2A_{i}\left(\left|\nu_{i}\left(s\right)\right|+\left|{\dot{\nu }}_{i}\left(s\right)\right|\right)\left|\nu_{i}\left(s\right)\right|\left.\left[\sum_{j=1}^{n}\left|a_{ij}\right|{\bar{f}}_{j}\left|+I_{i}\right|\right]\right\}ds\\ +2\sum_{i=1}^{n}\int_{0}^{t}e^{\varepsilon s}\sum_{j=1}^{n}c_{ij}\left(\nu_{i}\left(s\right)+{\dot{\nu }}_{i}\left(s\right)\right)\left(g_{j}\left(y_{j}\left(s\right)\right)-g_{j}\left(x_{j}\left(s\right)\right)\right)dB_{i}\left(s\right)\\ =V\left(0\right)+\sum_{i=1}^{n}\int_{0}^{t}e^{\varepsilon s}\left\{\left[2\varepsilon -2\pi_{i}+\left|\varepsilon +2-\gamma_{i}-\pi_{i}\right|+3{\bar{k}}_{i}\right.\right.\\ +{\bar{\alpha }}_{i}\sum_{j=1}^{n}\left|a_{ij}\right|l_{j}+3A_{i}\left.\left(\sum_{j=1}^{n}\left|a_{ij}\right|{\bar{f}}_{j}\left|+I_{i}\right|\right)\right]\nu_{i}^{2}\left(s\right)\\ +\left[\varepsilon +2-\right.2\gamma_{i}+\left|\varepsilon +2-\gamma_{i}-\pi_{i}\right|+{\bar{k}}_{i}+\sum_{j=1}^{n}{\bar{\alpha }}_{j}\left|a_{ji}\right|l_{i}\\ +\sum_{j=1}^{n}{\bar{\alpha }}_{i}\left|a_{ij}\right|l_{j}+A_{i}\left.\left.\left(\sum_{j=1}^{n}\left|a_{ij}\right|{\bar{f}}_{j}\left|+I_{i}\right|\right)\right]\nu_{i}^{2}\left(s\right)\right\}ds\\ +2\sum_{i=1}^{n}\int_{0}^{t}e^{\varepsilon s}\sum_{j=1}^{n}c_{ij}\left(v_{i}\left(s\right)+{\dot{v}}_{i}\left(s\right)\right)\left(g_{j}\left(y_{j}\left(s\right)\right)-g_{j}\left(x_{j}\left(s\right)\right)\right)\text{d}B_{i}\left(s\right). \end{array}$$

According to conditions in the theorem, there exits *ε* > 0 which satisfy

(44) $$\begin{array}{c} 2\varepsilon -2\pi_{i}+\left|\varepsilon +2-\gamma_{i}-\pi_{i}\right|+3{\bar{k}}_{i}+{\bar{\alpha }}_{i}\sum_{j=1}^{n}\left|a_{ij}\right|l_{j}+3A_{i}\left(\sum_{j=1}^{n}\left|a_{ij}\right|{\bar{f}}_{j}+I_{i}\right)\leq 0,\\ \varepsilon +2-2\gamma_{i}+\left|2-\gamma_{i}-\pi_{i}\right|+{\bar{k}}_{i}+\sum_{j=1}^{n}{\bar{\alpha }}_{j}\left|a_{ji}\right|l_{i}+\sum_{j=1}^{n}{\bar{\alpha }}_{i}\left|a_{ij}\right|l_{j}+A_{i}\left(\sum_{j=1}^{n}\left|a_{ij}\right|{\bar{f}}_{j}+I_{i}\right)\leq 0. \end{array}$$

Derive from (14) that

(45) $$\begin{array}{c} V\left(t\right)\leq \sum_{i=1}^{n}\left[\nu_{i}^{2}\left(0\right)+{\left(\nu_{i}\left(t\right)+{\dot{\nu }}_{i}\left(0\right)\right)}^{2}\right]\\ +2\sum_{i=1}^{n}\int_{0}^{t}e^{\varepsilon s}\sum_{j=1}^{n}c_{ij}\left(v_{i}\left(s\right)+{\dot{v}}_{i}\left(s\right)\right)\left(g_{j}\left(y_{j}\left(s\right)\right)-g_{j}\left(x_{j}\left(s\right)\right)\right)\text{d}B_{i}\left(s\right). \end{array}$$

Then,

(46) $$\begin{array}{c} \sum_{i=1}^{n}\left[\nu_{i}^{2}\left(t\right)+{\left(\nu_{i}\left(t\right)+{\dot{\nu }}_{i}\left(t\right)\right)}^{2}\right]\leq C_{0}e^{-\varepsilon t}+2\sum_{i=1}^{n}\int_{0}^{t}e^{\varepsilon \left(s-t\right)}\sum_{j=1}^{n}c_{ij}\left(\nu_{i}\left(s\right)+{\dot{\nu }}_{i}\left(s\right)\right)\\ \left(g_{j}\left(y_{j}\left(s\right)\right)-g_{j}\left(x_{j}\left(s\right)\right)\right)dB_{i}\left(s\right). \end{array}$$

Taking expectation of it,

(47) $$\begin{array}{c} \sum_{i=1}^{n}E\left[\nu_{i}^{2}\left(t\right)+{\left(\nu_{i}\left(t\right)+{\dot{\nu }}_{i}\left(t\right)\right)}^{2}\right]\leq e^{-\varepsilon t}E\left(C_{0}\right). \end{array}$$

Then,

(48) $$\begin{array}{c} \sum_{i=1}^{n}E\left[{\left(y_{i}\left(t\right)-x_{i}\left(t\right)\right)}^{2}\right]\leq e^{-\varepsilon t}E\left(C_{0}\right). \end{array}$$

where *ε* > 0,

(49) $$\begin{array}{c} C_{0}=\sum_{i=1}^{n}\left[{\left(\psi_{y_{i}}\left(0\right)-\psi_{x_{i}}\left(0\right)\right)}^{2}+{\left(\psi_{y_{i}}\left(0\right)-\psi_{x_{i}}\left(0\right)+\chi_{y_{i}}\left(0\right)-\chi_{x_{i}}\left(0\right)\right)}^{2}\right]. \end{array}$$

According to Definition 1, system (1) and system (3) are ES under control strategy *u*(*t*).

## 4. Numerical Examples

In this section, two examples are given to illustrate the theorems.

The CGSNNI is considered as follows:

(50) $$\begin{array}{c} d\left({\dot{x}}_{i}\left(t\right)\right)=-\gamma_{i}{\dot{x}}_{i}\left(t\right)dt-\alpha_{i}\left(x_{i}\left(t\right)\right)\left[h_{i}\left(x_{i}\left(t\right)\right)-\sum_{j=1}^{2}a_{ij}f_{j}\left(x_{j}\left(t\right)\right)-I_{i}\left(t\right)\right]dt\\ +\sum_{i=1}^{2}c_{ij}g_{j}\left(x_{j}\left(t\right)\right)dB_{i}\left(t\right),i=1,2. \end{array}$$

The corresponding slave system is as follows:

(51) $$\begin{array}{c} d\left({\dot{y}}_{i}\left(t\right)\right)=-\gamma_{i}{\dot{y}}_{i}\left(t\right)dt-\alpha_{i}\left(y_{i}\left(t\right)\right)\left[h_{i}\left(y_{i}\left(t\right)\right)-\sum_{j=1}^{2}a_{ij}f_{j}\left(y_{j}\left(t\right)\right)-I_{i}\left(t\right)\right]dt\\ +u_{i}\left(t\right)dt+\sum_{i=1}^{2}c_{ij}g_{j}\left(y_{j}\left(t\right)\right)dB_{i}\left(t\right),i=1,2. \end{array}$$

The control strategy is given as follows: *u*_*i*_(*t*)=−*π*_*i*_(*y*_*i*_(*t*) − *x*_*i*_(*t*)), *π*_*i*_ > 0, *i*=1,2.

**Example 1 .**

Let the parameters and the functions in system Example 1 be

(52) $$\begin{array}{c} \gamma_{1}=0.8,\gamma_{2}=1.1,a_{11}=0.3,a_{12}=0.5,a_{21}=-0.4,a_{22}=0.15. \end{array}$$

(53) $$\begin{array}{c} f_{j}\left(x_{j}\left(t\right)\right)=\sin\left(x_{j}\left(t\right)\right),g_{j}\left(x_{j}\left(t\right)\right)=\cos\left(x_{j}\left(t\right)\right),I_{i}\left(t\right)=e^{-t},i,j=1,2,\\ \pi_{1}=1.25,\pi_{2}=1.49,h_{1}\left(x_{1}\right)=2.6x_{1},h_{2}\left(x_{2}\right)=6x_{2}. \end{array}$$

*α*_1_(*x*_1_)=1/100(2+1/1+*x*_1_^2^) and *α*_2_(*x*_2_)=1/100(2 − 1/1+*x*_2_^2^). After calculating, one has

(54) $$\begin{array}{c} \underline{\alpha_{1}}=0.02,{\bar{\alpha }}_{1}=0.03,\underline{\alpha_{2}}=0.01,{\bar{\alpha }}_{2}=0.02,A_{1}=A_{2}=0.01,\\ {\bar{f}}_{j}=l_{j}={\bar{I}}_{i}=1,i,j=1,2,\underline{k_{1}}=0.048,{\bar{k}}_{1}=0.078,\underline{k_{2}}=0.11,{\bar{k}}_{2}=0.1125. \end{array}$$

One can see that assumptions (*H*_1_) − (*H*_3_) are satisfied and

(55) $$\begin{array}{c} p_{1}=2\eta_{1}-\gamma_{1}\eta_{1}-\left|1+\eta_{1}^{2}-\pi_{1}\right|-{\bar{k}}_{1}-A_{1}\sum_{j=1}^{2}\left|a_{1j}\right|{\bar{f}}_{j}-A_{1}I_{1}\\ -\sum_{j=1}^{2}{\bar{\alpha }}_{j}\left|a_{j1}\right|l_{1}-\sum_{k=1}^{2}\sum_{j=1}^{2}c_{kj}^{2}m_{1}^{2}=0.0555>0,\\ p_{2}=2\eta_{2}-\gamma_{2}\eta_{2}-\left|1+\eta_{2}^{2}-\pi_{2}\right|-{\bar{k}}_{2}-A_{2}\sum_{j=1}^{2}\left|a_{2j}\right|{\bar{f}}_{j}-A_{2}I_{2}\\ -\sum_{j=1}^{2}{\bar{\alpha }}_{j}\left|a_{j2}\right|l_{2}-\sum_{k=1}^{2}\sum_{j=1}^{2}c_{kj}^{2}m_{2}^{2}=1.496>0,q_{1}=2\left(\gamma_{1}-\eta_{1}\right)-\gamma_{1}\eta_{1}-\left|1+\eta_{1}^{2}-\pi_{1}\right|-{\bar{k}}_{1}-A_{1}\sum_{j=1}^{2}\left|a_{1j}\right|{\bar{f}}_{j}-A_{1}I_{1}\\ -\sum_{j=1}^{2}{\bar{\alpha }}_{j}\left|a_{1j}\right|l_{j}=0.1905>0,\\ q_{2}=2\left(\gamma_{2}-\eta_{2}\right)-\gamma_{2}\eta_{2}-\left|1+\eta_{2}^{2}-\pi_{2}\right|-{\bar{k}}_{2}-A_{2}\sum_{j=1}^{2}\left|a_{2j}\right|{\bar{f}}_{j}-A_{2}I_{2}\\ -\sum_{j=1}^{2}{\bar{\alpha }}_{j}\left|a_{2j}\right|l_{j}=0.606>0, \end{array}$$

which satisfy Theorem 1. Therefore, system (50) and system (51) are ES.

On the other hand, let the initial conditions be

(56) $$\begin{array}{c} \left[x_{1}\left(0\right),{\dot{x}}_{1}\left(0\right),y_{1}\left(0\right),{\dot{y}}_{1}\left(0\right)\right]=\left[1,0.3,-0.2,0.5\right];\\ \left[x_{2}\left(0\right),{\dot{x}}_{2}\left(0\right),y_{2}\left(0\right),{\dot{y}}_{2}\left(0\right)\right]=\left[0.9,0.6,0.3,0.7\right]. \end{array}$$

According to the simulation, one can see the instant response and the synchronization of the state variable in the drive system and the slave system in Example 1 (Figures 1–3).

Obviously, the simulation and Theorem 1 are consistent.

**Example 2 .**

Let the parameters and the functions in system Example 1 be *γ*_1_=2.1 and *γ*_2_=2.2.

Others parameters and functions are the same as Example 1. One sees that

(57) $$\begin{array}{c} 2\pi_{1}-\left|2-\gamma_{1}-\pi_{1}\right|-3{\bar{k}}_{1}-{\bar{\alpha }}_{1}\sum_{j=1}^{2}\left|a_{1j}\right|l_{j}-3A_{1}\left(\sum_{j=1}^{2}\left|a_{1j}\right|{\bar{f}}_{j}+I_{1}\right)=0.598>0,\\ 2\pi_{2}-\left|2-\gamma_{2}-\pi_{2}\right|-3{\bar{k}}_{2}-{\bar{\alpha }}_{2}\sum_{j=1}^{2}\left|a_{2j}\right|l_{j}-3A_{2}\left(\sum_{j=1}^{2}\left|a_{2j}\right|{\bar{f}}_{j}+I_{2}\right)=0.918>0,\\ 2\gamma_{1}-2-\left|2-\gamma_{1}-\pi_{1}\right|-{\bar{k}}_{1}-\sum_{j=1}^{2}{\bar{\alpha }}_{j}\left|a_{j1}\right|l_{1}-\sum_{j=1}^{2}{\bar{\alpha }}_{1}\left|a_{1j}\right|l_{j}-A_{1}\left(\sum_{j=1}^{2}\left|a_{1j}\right|{\bar{f}}_{j}+I_{1}\right)=0.435>0,\\ 2\gamma_{2}-2-\left|2-\gamma_{2}-\pi_{2}\right|-{\bar{k}}_{2}-\sum_{j=1}^{2}{\bar{\alpha }}_{j}\left|a_{j2}\right|l_{2}-\sum_{j=1}^{2}{\bar{\alpha }}_{2}\left|a_{2j}\right|l_{j}-A_{2}\left(\sum_{j=1}^{2}\left|a_{2j}\right|{\bar{f}}_{j}+I_{2}\right)=0.5725>0, \end{array}$$

which satisfy Theorem 2. Therefore, system (50) and system (51) are ES.

On the other hand, let the initial conditions be

(58) $$\begin{array}{c} \left[x_{1}\left(0\right),{\dot{x}}_{1}\left(0\right),y_{1}\left(0\right),{\dot{y}}_{1}\left(0\right)\right]=\left[2,0.3,0.7,0.5\right];\\ \left[x_{2}\left(0\right),{\dot{x}}_{2}\left(0\right),y_{2}\left(0\right),{\dot{y}}_{2}\left(0\right)\right]=\left[1,0.4,0.6,0.7\right]. \end{array}$$

According to the simulation, one can see the track of the instant response and the synchronization error of Example 2 (Figuers 4–6).

Obviously, the simulation is consistent with Theorem 2.

## 5. Conclusions

The ES of CGSNNI is studied in this paper. According to the definition of synchronization, there is an error system by the drive system and the slave one. Proper substitution of variable is used to transform the second-order system into a first one. In Theorem 1, properties of $i\hat{t}o$ integral, differential operator, and the second Lyapunov method are used to get a sufficient condition for the ES. In Theorem 2, the properties of calculus are used on the second-order differential equation to get a sufficient condition of exponential synchronization. At last, two examples are given to illustrate the theorems. The conditions in two theorems are different and can complement each other. They are different ways to decide if there is synchronization between the drive system and the slave system. In the examples simulated, Theorem 1 is suitable for Example 1 but not suitable for Example 2. Theorem 2 is suitable for Example 2 but not suitable for Example 1. The effectiveness of the theorems is verified. They provide two different ways. In application, we can choose one of them according to the parameters given in the system. Also, the method we used in the proof of two theorems can be adopted in other models with inertial terms and stochastic terms.

## Figures and Tables

**Figure 1:** The state of the drive variable 1 and the response variable 1 in example 1.

**Figure 2:** The state of the drive variable 2 and the response variable 2 in example 1.

**Figure 3:** The state of the error variable 1 and the error variable 2 in example 1.

**Figure 4:** The state of the drive variable 1 and the response variable 1 in example 2.

**Figure 5:** The state of the drive variable 2 and the response variable 2 in example 2.

**Figure 6:** The state of the error variable 1 and the error variable 2 in example 2.

## Data Availability

No data were used to support this study.
